# Extracts from Myrtle Liqueur Processing Waste Modulate Stem Cells Pluripotency under Stressing Conditions

**DOI:** 10.1155/2019/5641034

**Published:** 2019-06-11

**Authors:** Sara Cruciani, Sara Santaniello, Angela Fadda, Luana Sale, Giorgia Sarais, Daniele Sanna, Maurizio Mulas, Giorgio Carlo Ginesu, Maria Laura Cossu, Pier Andrea Serra, Carlo Ventura, Margherita Maioli

**Affiliations:** ^1^Department of Biomedical Sciences, University of Sassari, Viale San Pietro 43/B, 07100 Sassari, Italy; ^2^Laboratory of Molecular Biology and Stem Cell Engineering, National Institute of Biostructures and Biosystems–Eldor Lab, Innovation Accelerator, CNR, Via Piero Gobetti 101, 40129 Bologna, Italy; ^3^Instituto di Scienze delle Produzioni Alimentari (ISPA), Consiglio Nazionale delle Ricerche (CNR), Traversa la Crucca 3, 07100 Sassari, Italy; ^4^Department of Agriculture, University of Sassari, Via De Nicola 9, 07100 Sassari, Italy; ^5^Department of Life and Environmental Sciences, University of Cagliari, Via Ospedale 72, 09124 Cagliari, Italy; ^6^Institute of Biomolecular Chemistry (ICB), Consiglio Nazionale delle Ricerche (CNR), Traversa la Crucca 3, 07100 Sassari, Italy; ^7^General Surgery Unit 2 “Clinica Chirurgica” Medical, Surgical and Experimental Sciences Department, University of Sassari, Viale San Pietro 8, 07100 Sassari, Italy; ^8^Department of Clinical and Experimental Medicine, University of Sassari, Viale S. Pietro 43/b, 07100 Sassari, Italy; ^9^Department of Biomedical Sciences, Center for Developmental Biology and Reprogramming (CEDEBIOR), University of Sassari, Viale San Pietro 43/B, 07100 Sassari, Italy; ^10^Istituto di Ricerca Genetica e Biomedica, Consiglio Nazionale delle Ricerche (CNR), Monserrato, Cagliari, Italy

## Abstract

Nutraceuticals present in food are molecules able to exert biological activity for the prevention and treatment of various diseases, in form of pharmaceutical preparations, such as capsules, cream, or pills.* Myrtus communis *L. is a spontaneous Mediterranean evergreen shrub, widely known for the liqueur obtained from its berries rich in phytochemicals such as tannins and flavonoids. In the present study, we aimed to evaluate the properties of myrtle byproducts, residual of the industrial liqueur processing, in Adipose-derived stem cells (ADSCs) induced at oxidative stress by in vitro H_2_O_2_ treatment. Cells were exposed for 12-24 and 48h at treatment with extracts and then senescence-induced. ROS production was then determined. The real-time PCR was performed to evaluate the expression of inflammatory cytokines and sirtuin-dependent epigenetic changes, as well the modifications in terms of stem cell pluripotency. The *β*-galactosidase assay was conducted to analyze stem cell senescence after treatment. Our results show that industrial myrtle byproducts retain a high antioxidant and antisenescence activity, protecting cells from oxidative stress damages. The results obtained suggest that residues from myrtle liqueur production could be used as resource in formulation of food supplements or pharmaceutical preparations with antioxidant, antiaging, and anti-inflammatory activity.

## 1. Introduction

Nutraceuticals can be defined as a branch of biomedical science based on the biological action of specific molecules, which are part of food [1]. The officinal plants, described also as medicinal, have long been studied for their antiseptic, antibacterial, and anti-inflammatory properties [2]. They are also useful in the presence of allergies or diseases of the respiratory system and for cutaneous local treatment, for example, in case of psoriasis, eczema, and sunburn, thus performing protective action against various diseases [3, 4].

In recent years, the attention of researchers has been addressed to the study and the use of medicinal plants in clinical practice [5], thanks to their special antioxidant properties, cell cycle inhibition, promotion of tissue regeneration, and inhibition of acute inflammation [6, 7]. The role of free radical reactions, in fact, is well known for some pathologies.

Deregulation of reactive oxygen species (ROS) balancing is a key event during the onset and progression of pathological conditions related to aging, as cancer, diabetes, atherosclerosis, neurodegeneration, and inflammatory diseases [8–10]. Currently, it is also believed that even prooxidant agents or processes may exert a role in cell homeostasis, by stimulating the antioxidant defense system in cells and tissues, the so-called “oxidative stress preconditioning” or hormesis [11]. The term hormesis indicates an agent exerting a biphasic effect: at low doses representing a stimulus, while being toxic at high doses [12].

Recently, the development of nutraceuticals has become a great issue also applied to regenerative medicine. Regenerative medicine is based on the capability of stem cells to repair tissue damage and restore cellular homeostasis, by substituting damaged elements [13]. Although bone marrow has been used as the main source of hMSCs (hBMSCs), bone marrow collection remains a relatively invasive and painful procedure. Furthermore, the use of hBMSCs is potentially associated with a high degree of viral infection and a significant decline in cell viability and differentiation with donor age [14]. An ideal hMSCs source should allow the isolation of large amount of stem cells, collected with a minimally invasive procedure, and provide a hMSCs population maintaining good vitality and differentiating potential with donor's age [15, 16]. Adipose tissue represents a great source of stem cells, called Adipose-derived stem cells (ADSCs) [17], usually considered wasting material. hADSCs exhibit phenotypic and gene expression profiles similar to hMSCs obtained from bone marrow [18–20] and, under chemical and physical stimuli, are able to acquire different phenotypes, thus participating in tissue regenerative process [21–23]. Within this context, we have previously demonstrated that vitamin D together with melatonin exerts an important role in orchestrating stem cell fate [24] through activation of HDAC and sirtuins [25]. Moreover, other different natural molecules have been previously used by our group to achieve a specific cellular phenotype from human stem cells obtained from different sources [26, 27] or to control cell proliferation in hepatocarcinoma cells [28]. Another important key point in regenerative medicine is the loss of regenerative potential of stem cells during aging [29], which is deeply related to cellular senescence and ROS production [30]. Within these contexts, finding a natural product able to counteract senescence in stem cells and restore their regenerative potential could have a great impact in the interventions for age-related diseases. Berries of* Myrtus communis *L. (Myrtaceae), an evergreen spontaneous shrub, typical of the Mediterranean areas, contain a large amount of bioactive polyphenols [31, 32], mainly anthocyanins [33–35], and have long been known for anti-inflammatory, antiseptic, and antimicrobial properties [36]. In Sardinia,* Myrtus communis *is commonly used in the food industry, for the production of sweet liqueur obtained by hydroalcoholic extraction of the berries [37], to which follows the production of large quantities of residues (about 30.000 Kg/year) and waste material. The use of these biomasses is still limited being underexploited as compost for agricultural purposes. However, they represent large potential resources for use as food supplements, food additives, or as a raw material for the preparation of extracts with antimicrobial activity [38].

The aim of the present study was to analyze the effect of myrtle extracts on the molecular pathway controlling ADSCs senescence, obtained by H_2_O_2_ exposure in vitro. The use of these residues in medicine could represent large alternative resources in the cosmetic and pharmacological industry, to be used for the treatment of various diseases [39].

## 2. Materials and Methods

### 2.1. Biomass Collection

The biomasses of myrtle (byproducts), residual of the preparation of the homonymous liqueur, were used in this study. The industrial byproducts, kindly provided by a distillery located in Sardinia, were obtained after a process of infusion of the myrtle berries in hydroalcoholic solution for about 30 days. At the end of the infusion period, the berries were pressed and left to dry at room temperature to remove residual alcohol. In order to mimic the industrial process, a small-scale infusion was carried out in laboratory. With this purpose, berries belonging to 8 myrtle cultivars were harvested at maturity at the experimental orchard located in the “Antonio Milella” station of the University of Sassari (central western Sardinia, Italy) and mixed together with the aim of providing a uniform sample like that of the industrial supply. According to the industrial process, 200 g of berries was mixed with 750 mL of a hydroalcoholic solution (70% v/v) and stored for 30 days at room temperature (20°C) in dark bottles. At the end of the infusion period, the byproducts were separated from the hydroalcoholic extract, pressed, and freeze-dried. Once lyophilized, pulp and seeds were separated. The pulp of the industrial byproducts and that of the byproducts obtained in laboratory were used to prepare the extracts.

#### 2.1.1. Chemicals

All reagents and solvents used in this process were of analytical grade, unless otherwise specified and used without further purification. 2,2-Diphenyl-1-picryhydrazyl radical (DPPH) was purchased from Alfa Aesar (London, UK). 5,5-Dimethyl-1-pyrroline-N-oxide (DMPO) was purchased from Enzo Life Sciences.

### 2.2. Preparation and Characterization of Myrtus Extracts

#### 2.2.1. Preparation of Plant Extracts

Two grams of freeze-dried myrtle pulp byproducts were extracted twice with 40 mL of a methanol/water solution (70% MeOH) and sonicated in an ultrasonic cleaner (VWR International, Leuven, Belgium) for 1 hour at 25°C. The mixtures were centrifuged at 3000x g for 10 minutes. The organic extracts were filtered with Whatman 4 filter paper, evaporated to dryness under a nitrogen flow to remove methanol, and then freeze-dried to remove water. The freeze-dried extracts were used to assess the hydroxyl radical scavenging activity and the subsequent tests in vitro on stem cells.

### 2.3. Radical Scavenging Activity

#### 2.3.1. DPPH Radical Scavenging Activity

The DPPH radical scavenging activity was determined spectrophotometrically according to Fadda et al., 2014 [40]. The water extract properly diluted was mixed to 100*μ*L of DPPH (1 mM in absolute ethanol). The mixture was stored in the dark at room temperature for 1 h and UV-Vis-VIS readings were carried out with a spectrophotometer Agilent 8453 at 517 nm. The antiradical activity was expressed as TEAC units (mmols trolox/g of DW) using a Trolox calibration curve (5-20 *μ*M, R^2^ = 0.99).

#### 2.3.2. Hydroxyl Radical Scavenging Activity

The hydroxyl radical scavenging activity was determined with the spin trapping method coupled with Electron Paramagnetic Resonance (EPR) spectroscopy. The hydroxyl radicals were generated by Fenton reaction and trapped with a nitrone spin trap DMPO obtaining a DMPO-OH adduct [41]. In the Fenton reaction, iron(II) is oxidized by hydrogen peroxide to iron(III) generating a hydroxyl radical and a hydroxide ion. Before the analysis, the freeze-dried extracts were mixed with water in order to get the final concentration of 15 mg mL^−1^. The water extract, properly diluted, was mixed with 0.1 mM iron(II) sulfate, DMPO 26 mM, and hydrogen peroxide 0.03% (w/w) to a final volume of 1 mL with water. The DMPO adduct was detected with a Bruker EMX spectrometer operating at the X-band (9.4 GHz) using a Bruker Aqua-X capillary cell. EPR instrument was set under the following conditions: modulation frequency, 100 kHz; modulation amplitude, 1 G; receiver gain, 1 x 10^5^; and microwave power, 20 mW. EPR spectra were recorded at room temperature immediately after the preparation of the reaction mixture. The concentration of the DMPO-OH adduct was estimated from the double integration of spectra. The percentage of inhibition was calculated against a blank with no extract applying the following formula:

(1) $$\begin{array}{c} 100\times \frac{\left(A_{0}-A_{s}\right)}{A_{0}} \end{array}$$

where A_0_ is the concentration of the spin adduct without extract and A_s_ is the concentration of the adduct after the reaction with the extract. Results were expressed as EC_50_. Three replications were performed for each extract.

### 2.4. Cell Culturing and Treatment

ADSCs of human adult subcutaneous adipose tissue were obtained from male and female patients, during surgery processes (n=12, age=45± 15 years, BMI: 22 ± 3 kg/m2), after signing a written informed consent. Ethics Committee Review Boards for Human Studies in Sassari approved the study (n_ETIC 240I/CE 26 July 2016, Ethical committee, ASL Sassari). The samples collected were processed and the cells were isolated and characterized as previously described [24]. Cells at passage 5 were cultured in a basic growing medium composed of Dulbecco's modified Eagle's Medium (DMEM, Life Technologies, USA), 20% fetal bovine serum (FBS, Life Technologies, USA), 200 mM L-glutamine (Euroclone, Italy), and 200 U/mL penicillin−0.1 mg/mL streptomycin (Euroclone, Milano, Italy). To perform the tests in vitro, the freeze-dried* Myrtus* extracts was suspended in cultured medium at a final concentration of 0,5 mg/ml, derived from previously tests (data not shown), and then used directly in cell culture, for 12-24 and 48h. Cells used as control are cultured in the growing medium only. To induce senescence, after treatment with the extracts, cells were incubated for 1h with 100 *μ*M H_2_O_2_ in basic growing medium. For positive control of antioxidant activity and stressful conditions, ADSCs were cultured in the same conditions with 100 *μ*g/ml ascorbic acid (Sigma-Aldrich, Germany), known for its properties in regulation of immune system and chronic inflammation [42].

### 2.5. MTT Viability Assay

Cellular metabolic activity was evaluated by the Thiazolyl Blue Tetrazolium Bromide (MTT) assay (Sigma-Aldrich, Germany). Cells, cultured in the presence or absence of M*yrtus* extracts, in which senescence was induced as previously described, were seeded at a concentration of 10,000 cells/well in 96-well plates. After the attachment, cells were incubated with 200 *μ*l of different extracts for 12, 24, and 48 hours and then induced to senescence with H_2_O_2_. The medium was removed and 100 *μ*l MTT at final concentration of 0.65 mg/ml was added in each well and incubated for 2h. After incubation, formazan was dissolved in DMSO and absorbance detected at 570 nm using Varian50 MPR, Microplate reader. The viability of H2O2-senescenct cells precultured with M*yrtus* extracts (treated cells) was calculated as % cell viability referred to untreated control cells = (OD570 treated cells) × 100/(OD570 control).

### 2.6. SA-*β*-Gal Staining

To identify senescent cells in culture, “The Senescence Cells Histochemical Staining Kit” (Sigma-Aldrich, Germany) was used. ADSCs in 6-well plate are cultured for 12-24-48h in the presence or absence of* Myrtus* extracts and then induced to senescence with H_2_O_2_. At the end of the incubation time, the medium containing H_2_O_2_ was removed and the cells were fixed and processed according to the manufacturer's instructions. For evaluation of SA-*β*-Gal activity, cells were then observed by light microscopy. The number of positively blue-stained cells was calculated as the percentage of total number of cells.

### 2.7. Measuring of Nitric Oxide Production

To test the variation in nitric oxide (NO) production by the cells at different time points, Griess Reagent Kit for Nitrite Determination (Thermo Fisher Scientific, USA) was used. According to the manufacturer's instructions, 150 *μ*l of nitrite standard solution was added to each well of 96-well plate and incubated for 30 minutes. The nitrite concentrations were read as the absorbance at 548 nm wavelength of the nitrite-containing samples in a spectrophotometric microplate reader.

### 2.8. Gene Expression Analysis of Real-Time PCR

Total mRNA was isolated at times 0, 12, 24, and 48 hours from cells treated in previously described conditions, at passage 5, and used for quantitative polymerase chain reaction. RNA extraction was performed using the ChargeSwitch total RNA Cell Kits (Life Technologies, Grand Island, NY, USA) and approximately 1*μ*g of total RNA was reverse-transcribed into cDNA using the Superscript Vilo cDNA synthesis kit (Life Technologies, USA), according to the manufacturer's protocol. Quantitative polymerase chain reaction was performed in triplicate under standard qRT-PCR conditions (50°C for 2 min, 95°C for 2 min, and then cycled at 95°C for 15 s, 55–59°C for 30 s, and 60°C for 1 min, for 40 cycles), according to the qRT-PCR protocol specified in the Platinum® Quantitative PCR SuperMix-UDG Kit, using a CFX Thermal Cycler (Bio-Rad) (Applied Biosystems). The total volume of each reaction was 25 *μ*L, composed by 2X SuperMix with SYBR Green I, 0.1 *μ*M of each primer, and 3 *μ*L cDNA generated from 1*μ*g of the total RNA template. Target Ct values were normalized on hGAPDH, considered as a reference gene, while the mRNA levels of ADSCs treated in different conditions were expressed as fold of change (2−∆∆Ct) relative to the mRNA levels observed in ADSCs at time 0, before starting treatment. Each experiment included a distilled water control.

The qRT-PCR analysis was performed for the following genes: octamer-binding transcription factor 4 (Oct-4); Sex determining region Y-box 2 (Sox2); Homeobox protein Nanog (NANOG); NAD-dependent deacetylase sirtuin-1 (SIRT1); Interleukin 6 (IL-6); Tumor necrosis factor alpha (TNF-*α*); and Heat Shock Protein 90b (Hsp90b). All primers were designed with Primer3, spanning all exons and highly specific. They are from Invitrogen and are described in Table 1.

### 2.9. Statistical Analysis

Statistical analysis was performed using Statistical Package for the Social Sciences version 13 Software (SPSS Inc., Chicago, IL, USA). The experiments were performed two times with three technical replicates for each treatment. The distributions of each group variance were evaluated with Kruskal-Wallis rank sum and Wilcoxon signed-rank test, assuming a p value <0.05 as statistically significant.

## 3. Results

### 3.1. Radical Scavenging Activity

Table 2 shows the hydroxyl and the DPPH radicals scavenging activities of myrtle byproducts. The DPPH radical scavenging activity of myrtle residues obtained from the industrial process was consistent with results of antiradical activity measured on fresh myrtle berries [43].

Both in industrial products and in fresh berries, the pulp, rich in anthocyanins and flavonoids, showed a high DPPH radical scavenging activity as compared to other plant species [44]. The hydroxyl radical scavenging activity, measured in the same extracts, confirmed the highest antiradical activity of the evaluated products. The hydroxyl radical (·OH) is one of the major causes of oxidative stress in living cells; its low selectivity makes this radical extremely reactive towards lipids, proteins, and nucleic acids [44, 45].

### 3.2. Myrtus Extract Regulates Cytokine Secretion in Inflammatory Response

Figure 1 shows the expression of proinflammatory cytokines Interleukin 6 (IL-6) (Figure 1(a)) and Tumor necrosis factor alpha (TNF-*α*) (Figure 1(b)) in cells exposed to* Myrtus* extracts for 12, 24, or 48h. IL-6 significantly decreased at 12h of treatment, compared to untreated cells, for all cultured conditions, including industrial byproduct, a sign that after industrial liqueur production the berries retain some of their properties. On the other hand, TNF-*α* is upregulated after 48h of extracts exposure, suggesting that* Myrtus* can counteract the inflammation induced by oxidative stress, but at the same time, it may promote tissue regeneration by cytokine secretion and stem cell recruitment.

### 3.3. Modulation of Nitric Oxide Production by Myrtus Treatment

*Myrtus* byproducts, both laboratory and industrial, have shown a potent antioxidant activity, decreasing significantly the nitric oxide (NO) production after induction of oxidative stress. This reduction was higher at 12 and 24h of treatment for both of* Myrtus* extracts, compared to untreated cells (Figure 2). The berries residual of liquor production have maintained their properties, exerting an important antioxidant response at stressor event.

### 3.4. Gene Expression Analysis of Pluripotency Related Genes

Exposure of ADSCs to laboratory and industrial byproducts revealed a significative upregulation of pluripotency related genes, Oct-4 (Figure 3(a)), Sox2 (Figure 3(b)), and NANOG (Figure 3(c)) compared to untreated cells, suggesting a promotion of regenerative potential of stem cells after stressful conditions. This overexpression of mRNA levels was already evident since the first hours of treatment, but reached its maximum after 48h.

### 3.5. The Antisenescent Effect of Myrtus Involves Sirtuin-Dependent Epigenetic Changes and Regulates the Expression of HSP

Figure 4 shows the capability of* Myrtus* extracts to induce SIRT1 activity with a significant increase in mRNA levels at 48h of treatment (panel (a)). Furthermore, treatment with M*yrtus* extracts has increased the levels of HSP90b (panel (b)), suggesting a role of this compound to protect cells from oxidative stress damage.

### 3.6. Effects of Myrtus on ADSCs Senescence-Induced by H_*2*_O_*2*_ Treatment

Consistent with previously described real-time PCR analysis, of protection from oxidative stress damages, Figure 5 shows the results from *β*-galactosidase staining assay, used to evaluate whether ADSCs treatment with* Myrtus* byproducts may oppose the premature senescence elicited by H_2_O_2_ treatment. Results have revealed that the extracts are able to significantly counteract the senescence process (panel (b)) and protect cells by oxidative stress damages. *β*-gal analysis at light microscope has revealed that both Lab and Ind by-P exert an antisenescence activity, that was higher for 24 and 48h of treatment, compared to untreated cells (panel (a)).

### 3.7. Myrtus Maintains Mitochondrial Activity in H_*2*_O_*2*_-Senescent ADSCs

The yellow tetrazolium salt is enzymatically converted into purple formazan precipitate in viable cells by mitochondrial succinate dehydrogenase. Our results showed that* Myrtus *extracts are able to preserve the mitochondrial activity and the viability of treated cells even after H_2_O_2_ exposure, for all different time-points, compared to the control untreated-senescent cells (Figure 6). Moreover, the waste industrial residues of* Myrtus* compounds are not cytotoxic for the cells, whose vitality is maintained, if not even increased, as compared to untreated controls not exposed to oxidative stress.

## 4. Discussion

The human body has the capability to cope with various environmental stresses, introducing adaptation mechanisms to restore the physiological balance. Altered functioning of biological processes is due to some pathological conditions such as aging, diabetes, atherosclerosis, and cancer [46]. In recent years, numerous studies have reported that natural molecules, like flavonoids and anthocyanins contained in food, show anticancer properties and protect against various diseases [47]. Some authors describe a significant cytotoxic effect of polyphenols on tumor cells with the inhibition of proliferation and consequent induction of apoptosis after treatment [48, 49].

Also flavonoids content in* P. macrocarpa* fruits have cytotoxic activities on different carcinoma cell lines, like human cervical, colon, and breast [50].

*Myrtus *is a spontaneous Mediterranean evergreen shrub used in the industrial field for the formulation of the liqueur [51], but it is also known for containing classes of biomolecules used as phytochemicals, including phenolic compounds such as tannins, quercetin, and gallic and ellagic acids in the seeds of its berry pulp [42, 50, 51]. As shown in Table 2, the laboratory and industrial byproducts used in this study have high radical scavenging activity, which depends on the percentage of anthocyanins, flavonoids, and tannins able to protect living cells from oxidative stress.

The molecules contained in myrtle berry are able to exert antimicrobic, anti-inflammatory, and antiaging activities and in particular are known for their free radical-scavenging activities, so they are used as a potent antioxidant [52]. Several in vitro studies have demonstrated that quercetin protects against oxidative damage and has a protective effect in stress-induced cells [53]. Extensive ROS production correlates with the loss of tissue homeostasis, leading to dysfunctional patterns, associated with inflammatory response [52, 53].

Inflammation is a frequently occurring response to several pathological conditions to protect tissue integrity against injuries, being also dangerous according to the dose and time of exposure [54, 55]. Oxidative stress induction with H_2_O_2_ treatment causes premature cellular senescence [56] and can activate an inflammatory response, associated with cytokine production [57]. Chemical components of Mediterranean plants, such as polyphenols, gallic acid derivatives, and flavonols, exert antioxidant and anti-inflammatory activity by inhibition of enzymes involved in ROS production [57, 58]. Polyphenols are capable of reducing ROS secretion and modulate the nitric oxide (NO) production and enzymatic activity involved in inflammatory response and cell activation, by downregulating TNF-*α* release and the levels of serological markers like IL-6 cytokine [56, 57]. Other authors described that treatment with* S. grandiflora* extracts decreased the level of IL-6 and TNF-*α* and colon inflammation in mice, related to ROS scavenging activity, and inhibitory action on inflammatory response [59]. Consistent with these studies*, Myrtus* extracts have shown a significative decrease in IL-6 expression at 12h of treatment, in cells cultured in the presence of Lab by-P, but also with Ind by-P, compared to H_2_O_2_-senescent ADSCs cultured in growing medium alone, demonstrating a potential anti-inflammatory effect of industrial waste materials (Figure 1(a)). The upregulation of IL6 and TNF-*α* (Figure 1(b)) suggests that* Myrtus* extracts may effectively counteract the inflammation induced by oxidative stress and at the same time promote tissue regeneration by stem cells recruitment. Inflammation in fact is an important response of the organisms after damage and plays an important role in tissue regeneration, through the secretion of TNF-*α* and IL-6 and in the presence of low ROS production [60]. Organisms possess a redox balance system able to modulate the cellular and tissue stress responses to maximize physiological defense processes [61]. High ROS production contributes to the development of many pathological conditions, proteins alteration, and activation of inflammatory acute response and premature cell senescence [62]. Phytochemicals and natural compounds can directly interact with nuclear receptors and enzymes of cell signaling, modulating natural antioxidant responses [59, 60]. Myrtle is described as able to exert antioxidant and anti-inflammatory activity in the treatment of different respiratory disorders, related to a fibrosis of the tissue and progressive loss of function [63]. The pretreatment for 12h-24h of H_2_O_2_-senescent ADSCs with different* Myrtus* byproducts has proved able to significantly decrease the NO production induced by H_2_O_2_-oxidative stress stimulation, compared to untreated cells (Figure 2).* Myrtus* extracts can, therefore, be considered involved in the activation of cell redox system, scavenging high amounts of ROS induced by oxidative stress and modulating the activity of enzymes recruited in antioxidant response and balancing.

A limited ROS production together with the modulation of TNF-*α* release plays a crucial role in stem cell recruitment in the sites of injuries, promoting cell migration and tissue regeneration [64]. Adipose-derived stem cells have self-renewal potential and can differentiate into different cell lineages, becoming adipocytes, chondrocytes, and osteocytes, representing an important resource in regenerative medicine [65]. In the present paper, ADSCs exposed to extracts, in particular Lab by-P, but also Ind by-P, showed a significant increase in mRNA levels of the principal markers of pluripotency, Oct-4, Sox2, and NANOG, as compared with untreated cells (Figure 3), suggesting that* Myrtus* berries have a high antioxidant activity and promote tissue regeneration after damage. This effect has also been previously shown by other authors, who describe an interesting circuit between SIRT1 and Nanog gene expression, modulated by ROS and p53 [66]. In the present paper, we show a similar gene expression trend between SIRT1 and Nanog after* Myrtus* extracts stimulation, reaching a maximum of their expression after 48 hours in culture (Figure 3).

Oct-4 is the main actor in stem cell pluripotency by suppressing molecular pathways of differentiation and by directly activating SIRT1 deacetylase. In actual fact, Oct-4 is correlated to the downregulation of SIRT1 and cell differentiation [67].

The NAD-dependent class III histone deacetylase sirtuin-1 (SIRT1) regulates various physiological processes and is involved in metabolism, stress response, and aging [68]. Some studies in vitro have demonstrated that inhibition of SIRT1 promotes the secretion of inflammatory cytokine, while, on the contrary, its overexpression prevents premature senescence [69]. Gene expression analysis in ADSCs treated with different* Myrtus* extracts (Lab by-P and Ind by-P) demonstrated that SIRT1 expression is upregulated starting from 12h of treatment, reaching a maximum after 24h-48h of treatment (Figure 4). This overexpression is strictly related to the prevention of premature senescence (Figure 5) and to a higher resistance to oxidative stress. *β*-gal analysis has revealed that both Lab and Ind by-P exert an antisenescence activity, in a time-dependent manner (higher for 24h and 48h of treatment), counteracting the premature ADSCs senescence, induced by H_2_O_2_ treatment, (Figure 5).

Our results demonstrate that* Myrtus* extracts have the capability to induce SIRT1 activity and prevent cell senescence in vitro in cells exposed to oxidative stress. Furthermore, phytochemicals are involved in Heat Shock-induced response as a mechanism for Self-Defense [70]. Heat Shock Proteins (HSPs) are mainly responsible for maintaining protein homeostasis and play an important role in aging [71].

Hsp90b is constitutively expressed in human cells, and its levels increased when cells are exposed to different kinds of stressors to maintain viability [72]. HSP inhibition associated with altered H_2_O_2_ balance leads to the generation of oxidative stress [73]. ADSCs treatment with* Myrtus* extracts has determined an increase in mRNA levels of Hsp90b (Figure 4(b)), which may suggest a role for this compound in stimulating the secretion of Hsp90b and protecting cells from oxidative stress damage.* Myrtus* industrial waste is able to protect the cells increasing their viability and maintaining their mitochondrial activity under stressing conditions (Figure 6).

## 5. Conclusions

Taken together, these results suggest that* Myrtus *have important antioxidant and protective activities to defend cells from stressful and harmful conditions, by epigenetically modulating HSP90b gene expression via SIRT1.

In addition, our findings demonstrate that* Myrtus* extracts can also have a regenerative potential by modulating stem cell pluripotency and inflammatory response. An intriguing observation suggests that the Ind by-P, residual of industrial production, maintains a large part of* Myrtus* properties and could be used as alternative resource in formulation of food supplements or cosmetics, as well as pharmaceutical preparations to be used for the treatment of various diseases.

## Figures and Tables

**Figure 1:** Expression of proinflammatory cytokines Il-6 and TNF-*α*. The expression of Interleukin 6 (IL-6) (a) and Tumor necrosis factor alpha (TNF-*α*) (b) was evaluated in H_2_O_2_-senescent ADSCs exposed for 12, 24, or 48h to ascorbic acid (CTRL+, blue bar) or to Lab by-P (yellow bar) or Ind by-P (red bar). The mRNA levels for each gene were expressed as fold of change (2−∆∆Ct) of mRNA levels observed in untreated ADSCs (CTRL-, black bar) defined as 1 (mean ±SD; n=6) and normalized to Glyceraldehyde-3-Phosphate-Dehidrogenase (GAPDH). Data are represented as mean± SD referring to the control (*∗*  p ≤ 0.05).

**Figure 2:** Measuring nitric oxide production after oxidative stress induction. The NO concentration was evaluated in ADSCs exposed for 12, 24, or 48h to ascorbic acid (CTRL+, blue bar), at Lab by-P (yellow bar), or at Ind by-P (red bar) and then induced to oxidative stress, compared to untreated H_2_O_2_-senescent cells (CTRL-, black bar). The nitrite concentrations were read as the absorbance at 548 nm for each sample and were expressed as mean± SD referring to the control (*∗*  p ≤ 0.05).

**Figure 3:** Expression of pluripotency related genes. The expression of octamer-binding transcription factor 4 (Oct-4) (a). Sex determining region Y-box 2 (Sox2) (b) and Homeobox protein Nanog (NANOG) (c) were evaluated in H_2_O_2_-senescent ADSCs exposed for 12, 24, or 48h to ascorbic acid (CTRL+, blue bar), at Lab by-P (yellow bar), or at Ind by-P (red bar). The mRNA levels for each gene were expressed as fold of change (2−∆∆Ct) of mRNA levels observed in untreated ADSCs (CTRL-, black bar) defined as 1 (mean ±SD; n=6) and normalized to Glyceraldehyde-3-Phosphate-Dehidrogenase (GAPDH). Data are represented as mean± SD referring to the control (*∗*  p ≤ 0.05).

**Figure 4:** Expression of Sirtuins and Heat Shock Proteins in ADSCs induced to oxidative stress. The expression of NAD-dependent deacetylase sirtuin-1 (SIRT1) (a) and Heat Shock Protein 90b (Hsp90B) (b) was evaluated in H_2_O_2_-senescent ADSCs exposed for 12, 24, or 48h to ascorbic acid (CTRL+, blue bar), to Lab by-P (yellow bar), or to Ind by-P (red bar). The mRNA levels for each gene were expressed as fold of change (2−∆∆Ct) of mRNA levels observed in untreated ADSCs (CTRL-, black bar) defined as 1 (mean ±SD; n=6) and normalized to Glyceraldehyde-3-Phosphate-Dehidrogenase (GAPDH). Data are represented as mean± SD referring to the control (*∗*  p ≤ 0.05).

**Figure 5:** Senescence-associated *β*-galactosidase activity. (a) *β*-galactosidase was evaluated in H_2_O_2_-senescent ADSCs treated with ascorbic acid (CTRL+), with Lab by-P, or with Ind by-P for 12, 24, or 48h, compared to untreated ADSCs (CTRL-). Scale bar=100 *μ*m. (b) The numbers of positive (blue) and negative cells were counted under the light microscope and the percentage of SA-*β*-Gal-positive cells for each treatment was calculated as the number of positive cells divided by the total number of cells counted using an image software analysis (ImageJ). Data are expressed as mean± SD referring to the control (*∗*  p ≤ 0.05).

**Figure 6:** Mtt assay of the ADSCs treated with* Myrtus* extracts related to the untreated cells (grey bar). Cell Viability = {OD570 of treated cells} × 100%/{OD570 of control cells, considered as 100}. The data were entered using SPSS Version 2.0 (IBM SPSS, 2013). Data are expressed as mean± SD referring to the control (*∗*  p ≤ 0.05).

**Table 1:** Primers sequences.

Primers	Forward	Reverse
hGAPDH	GAGTCAACGGAATTTGGTCGT	GACAAGCTTCCCGTTCTCAG
Oct-4	GAGGAGTCCCAGGCAATCAA	CATCGGCCTGTGTATATCCC
Sox2	CCGTTCATGTAGGTCTCGGAGCTG	CAACGGCAGCTACAGCTAGATGC
NANOG	CATGAGTGTGGATCCAGCT	CCTGAATAAGCAGATCCAT
SIRT1	CATTTTCCATGGCGCTGAGG	TGCTGGTGGAACAATTCCTGT
IL-6	TCTCAACCCCCAATAA	GCCGTCGAGGATGTA
TNF-*α*	CCTCAGACGCCACAT	GAGGGCTGATTAGAGAGA
Hsp90b	AGTTGGAATTCAGGGCATTG	TTTCTCGGGAGATGTTCAGG

**Table 2:** DPPH and hydroxyl radicals scavenging activities of *myrtle* byproducts obtained from the production of myrtle liqueur at industrial and laboratory level.

Antiradical activity	DPPH	Hydroxyl radical
	mmols trolox/g d.w.	EC50 (mg/mL)
Industrial byproducts	1,45 ± 0,01	0,48 ± 0,03
Laboratory byproducts		
Pulp	1,06 ± 0,2	0,64 ± 0,01

## Data Availability

The data used to support the findings of this study are included within the article.
